# The Efficacy of Hydroxychloroquine Combined with Huangqi Tablets in the Treatment of Diabetic Nephropathy

This article has been retracted.

**DOI:** 10.1155/2021/7988924

**Published:** 2021-10-18

**Authors:** Xiaorong Chen, Danhong Sheng, Xiangdong Kong

**Affiliations:** Department of Nephrology, the First People's Hospital of Fuyang Hangzhou, Hangzhou, Zhejiang 311400, China

## Abstract

**Objective:**

This study aimed to analyze the effect of hydroxychloroquine combined with Huangqi tablets in the treatment of diabetic nephropathy (DN).

**Methods:**

Eighty patients with DN were enrolled and divided into two groups by a random number table. 27 patients received routine treatment + hydroxychloroquine (group A), while 27 patients received routine treatment + hydroxychloroquine + Huangqi tablets (group B) and 26 patients received routine treatment (group C).

**Results:**

FPG, 2h PG, and HbA1c levels as well as TC and TG levels were lower in group B than in groups A and C at the end of 3 months of treatment and were lower in group A than in group C (*P* < 0.05). SCR, BUN, and 24-hour urine protein were reduced in group B after therapy, whereas eGFR was increased and the difference between groups A and C was significant (*P*=0.05). After treatment, VEGF, IGF-1, and TGF-1 levels were lower in group B than in groups A and C and in group A than in group C (*P*=0.05). Total symptom scores at 2, 4, and 6 months after treatment was lower in group B than in groups A and C, and they were lower in group A than in group C at all time points (*P* < 0.05). The total effective rates of treatment in groups A, B, and C were 66.67%, 88.89%, and 38.46% (*P* < 0.05). The incidence of adverse reactions in groups A, B, and C was 37.04%, 25.93%, and 11.54% (*P* > 0.05).

**Conclusion:**

Hydroxychloroquine combined with Huangqi tablets in the treatment of DN showed the best efficacy, with better control of blood glucose and lipids, which can more effectively delay the progression of renal lesions and effectively inhibit the expression of VEGF, IGF, and TGF-*β*1 in tethered cells with high safety.

## 1. Introduction

Diabetic nephropathy (DN) is a common complication of type 2 diabetes. If left untreated, it can lead to glomerulosclerosis, which can seriously increase the disability and mortality rates in patients with type 2 diabetes [1]. In addition, DN is considered to contribute to the occurrence of end-stage renal disease. In this case, patients may need to receive renal replacement therapy [2].

The early stage of DN will be manifested as microproteinuria, which can be reversed by effective treatment. However, if microalbuminuria keeps increasing, the condition will continue to worsen, causing edema and proteinuria and eventually renal failure [3]. Controlling blood glucose and blood pressure, as well as fat and protein consumption, is part of the current therapeutic therapy for DN. [4]. However, these treatments can only temporarily control the condition and have little effect on the progression of DN, and the prognosis of patients cannot be improved [5]. Hydroxychloroquine is a class of immunosuppressants widely used in the treatment of immuno-rheumatic diseases, and its efficacy was confirmed in immuno-rheumatic diseases [6]. It was thought that hydroxychloroquine had some therapeutic benefits in nephropathy, and cyclophosphamide with hydroxychloroquine had good outcomes in refractory nephrotic syndrome therapy [7]. Studies centered on hydroxychloroquine in the treatment of patients with nephropathy have found more prominent hypolipidemic, immunomodulatory, and antiplatelet effects [8].

However, it has also been found clinically that administration of hydroxychloroquine only is more pronounced, including gastrointestinal adverse effects, retinopathy, and central nervous system lesions [9]. To solve this problem, some scholars have proposed to combine the mild mechanism of action of herbals to moderate the toxic effects of Western drugs and enhance the safety of treatment [10]. As a result, the current research preanalyzed the therapeutic efficacy of hydroxychloroquine coupled with Huangqi pills in 80 patients with diabetic nephropathy described as follows.

## 2. Materials and Methods

### 2.1. Data

Eighty patients with DN in our hospital were selected. The inclusion criteria were age ≥18 years, meeting the diagnostic criteria for type 2 diabetes in the Chinese Guidelines for the Prevention and Treatment of Type 2 Diabetes (2017 edition) [11], meeting the diagnostic criteria for DN in the Clinical Diagnostic and Treatment Guidelines: The Chinese Medical Association's Nephrology Sub volume [12], urine protein volume of 1.0 g/24 h, blood creatinine of 133 umol/L, and fulfilling the Traditional Chinese Medicine criteria for qi and yin deficit and blood stasis blocking the collaterals. Exclusion criteria: patients with type 1 diabetes, gestational diabetes, comorbidities such as diabetic ketoacidosis and hyperosmolar coma, as well as those with severe cardiovascular and cerebrovascular diseases, those with other renal diseases such as IgA nephropathy, microscopic lesions, lupus nephritis, hepatitis B-associated nephritis, hypertensive kidney disease, purpura nephritis, individuals with acute and chronic infectious illnesses, severe exercise, autoimmune disorders, hematologic diseases, cancers, and mental problems, and those with medication allergies.

### 2.2. Methods

Group A was given routine treatment + hydroxychloroquine. Routine treatment included regular blood glucose control with oral hypoglycemic drugs or subcutaneous insulin injection to achieve fasting blood glucose <7.0 mmol/L and 2-hour postprandial blood glucose <11.1 mmol/L. Meanwhile, oral irbesartan (0.15 g^*∗*^7 s, J20130049, Sanofi Pharmaceuticals Co., Ltd.) 150 mg/d was given. For those with combined hypertension, to regulate blood pressure, angiotensin-converting enzyme inhibitors (ACEI) and angiotensin receptor blockers (ARBs) may be used to attain a systolic/diastolic blood pressure of 130/80 mmHg. In addition, hydroxychloroquine (0.1 g^*∗*^14 tablets, H19990263, Shanghai Central and Western Pharmaceutical Co., Ltd.) b.d 200 mg was given.

Group B was given routine treatment + hydroxychloroquine + Huangqi tablets. The routine treatment was the same as group A, hydroxychloroquine b.d 200 mg/time. Huangqi tablets (0.41 g^*∗*^36 s, Z20090313, Sichuan Chili Pharmaceutical Co., Ltd.) b.d. 4 tablets were given.

Group C received the same therapy as group A. All three groups were treated for three months and then followed up for another three months.

### 2.3. Outcome Measurement

Blood glucose: fasting blood glucose (FPG), 2-hour postprandial glucose (2h PG), and glycated hemoglobin (HbAlc) levels were measured in both groups before and 3 months after treatment. HbA1c levels were determined by the enzymatic method, and the glucose oxidase technique was used to detect FPG and 2-hour PG. All procedures were carried out in full accordance with the kit's instructions.

Lipids: total cholesterol (TC) and triglyceride (TG) levels were measured in both groups before and 3 months after treatment, respectively, using a fully automated biochemical analyzer. The TC and TG kits were selected to determine TC and TG levels by the enzymatic colorimetric method.

Renal function: blood creatinine (SCR), urea nitrogen (BUN), 24-hour urine protein, and estimated glomerular filtration rate (eGFR) were measured before and after treatment in both groups. SCR measurement: 5 ml of fasting venous blood was centrifuged at 3 000 r/min (*r* = 9 cm) for 10 min, and the supernatant was obtained and detected by a Hitachi 7600 automatic biochemical analyzer. BUN: morning urine was retained for determination by radioimmunoassay. 24-hour urine protein quantification: 24-hour urine was collected, and the volume was recorded and measured by the immunoturbidimetric method. eGFR was calculated according to the modified MDRD formula, i.e., eGFR = 186 × SCR−1.154 ×  age - 0.203 × (female × 0.742) × (China × 1.233).

Changes in the expression of vascular endothelial growth factor (VEGF), insulin-like growth factor-1 (IGF-1), and transforming growth factor 1 (TGF-1) in mesangial cells were evaluated using real-time fluorescence quantitative PCR and western blotting before and three months after therapy.

Symptom score [13]: symptoms included fatigue, shortness of breath and lazy speech, easy sweating, scaling skin, back and spine pain, mucous mouth and desire to drink, sphoria with feverish sensation in chest, palms and soles, dry throat and thirst, purplish dim tongue, and whitish glossy coating of the tongue. Each symptom was rated on a 0–4 scale. Level zero was no symptom, level 1 was mild symptom, level 2 was moderate symptom, and level 3 was severe symptom; the total symptom score ranges 0–30 points. The evaluation was performed once before treatment, 2 months, 4 months, and 6 months after treatment, respectively.

Efficacy criteria = reduction rate of symptom score = (pretreatment symptom score − posttreatment symptom score)/pretreatment symptom score^*∗*^100% [14]. Exceptionally effective: symptoms and signs vanished by the conclusion of therapy, SCR fell by more than 30%, and the patient's symptom score fell by more than 90%. Improvement: symptoms and signs improved at the end of treatment, SCR decreased by 5%–15%, and the patient's symptom score decreased by 30–89%. Ineffective: symptoms and signs were still obvious or even aggravated after the end of treatment, SCR decreased by less than 5%, and the patient's symptom score decreased by less than 30% [15]. Total effective rate = (number of patients with markedly effective + number of patients with improvement)/total number of cases^*∗*^100%.

Safety: the incidence of gastrointestinal adverse reactions, retinopathy, central nervous system lesions, dizziness, and creatinine elevation during treatment were compared between two groups.

### 2.4. Statistical Methods

Data were analyzed using SPSS 19.0 statistical software, and measures were expressed as mean ± standard deviation ($\bar{x}\pm s$), with *t*-test for comparison of means and chi-square test for comparison of rates. Figures were produced with GraphPad Prism 8. *P* < 0.05 indicated a significant difference.

## 3. Results

### 3.1. Baseline Data

There was no statistical difference in gender, mean age, mean body mass index (BMI), duration of type 2 diabetes, and duration of DN among groups A, B, and C (*P* > 0.05) (Table 1).

### 3.2. Blood Glucose

No significant differences in pretreatment FPG, 2h PG, and HbA1c levels were found in groups A, B, and C (*P* > 0.05). FPG, 2-hour PG, and HbA1c levels were lower in groups. They were substantially different in groups A and B after 3 months of therapy than before treatment (*P* 0.05), while they were not statistically different in group C before and after treatment (*P* > 0.05). FPG, 2-hour PG, and HbA1c levels were lower in group B than in groups A and C at the end of 3 months of treatment (*P* < 0.05), and all levels in groups A were lower than those of group C (*P* < 0.05) (Figure 1).

### 3.3. Blood Lipids

The differences in TC and TG levels before treatment among groups A, B, and C were not statistically significant (*P* > 0.05). After 3 months of treatment, TC and TG levels in groups A and B were lower before treatment (*P* < 0.05) and did not change significantly within group C (*P* > 0.05). TC and TG levels were lower in group B than in groups A and C at the end of 3 months of treatment (*P* < 0.05), and TC and TG levels of group A were lower than those of group C (*P* < 0.05) (Figure 2).

### 3.4. Renal Function

The differences in pretreatment SCR, BUN, 24-hour urine protein, and eGFR were not statistically significant among groups A, B, and C (*P* > 0.05). However, they were substantially lower in groups A and B after the three-month therapy period as compared to pretreatment values, and there was a significant increase in eGFR (*P* < 0.05), with no statistically significant difference before and after treatment in group C (*P* > 0.05). SCR, BUN, and 24-hour urine protein were lower in group B than in groups A and C after 3 months of treatment. Still, eGFR was higher than that in groups A and C (*P* < 0.05), and these indexes differ significantly between group A and group C after 3 months of treatment (*P* < 0.05) (Figure 3).

### 3.5. Cytokines

Before treatment, the differences in VEGF, IGF-1, and TGF-*β*1 levels in groups A, B, and C were not significant (*P* > 0.05). After treatment, VEGF, IGF-1, and TGF-*β*1 levels were lower in groups A and B than before treatment (*P* < 0.05). VEGF, IGF-1, and TGF-*β*1 levels were lower in group B after treatment than in groups A and C (*P* < 0.05), and these indexes in groups A were lower than those in group C after treatment (*P* < 0.05) (Figure 4).

### 3.6. Symptom Score

There was no significant difference in pretreatment symptom scores among groups A, B, and C (*P* > 0.05). After 2 months, 4 months, and 6 months of therapy, overall symptom ratings were lower in groups A and B (*P* 0.05), and the difference was statistically significant when comparing several periods (*P* 0.05). The difference in symptom scores did not differ significantly between before treatment and 2 months after treatment (*P* > 0.05), and the symptom score at 4 months and 6 months after treatment was lower than those before treatment (*P* < 0.05). The total symptom score at 2 months, 4 months, and 6 months after treatment in group B was lower than that in groups A and C and were lower in group A than in group C at all time points (*P* < 0.05) (Figure 5).

There was no significant difference in the pretreatment symptom score between groups A, B, and C (*P* > 0.05), which was lower in groups A and B at 2, 4, and 6 months after treatment compared with group C (*P* < 0.05). ^*∗*^*P* < 0.05.

### 3.7. The Total Effective Rate

The total effective rate in group A was 66.67% after 3 months of treatment, which was lower than the total effective rate in group B (88.89%) (*P* < 0.05), and the overall effective rate in both groups A and B (38.46%) was greater than that in group C (*P* 0.05) (Table 2).

### 3.8. Safety

The incidence of adverse reactions during treatment in group A was 37.04%, which was slightly higher than 25.93% of group B (*P* > 0.05), and the incidence of adverse reactions in both groups A and B was higher than that in group C (11.54%) (*P* < 0.05) (Table 3).

## 4. Discussion

Modern research has shown that the occurrence of DN correlated with combined factors such as genetics, hypertension, hyperglycemia, biochemical metabolic disorders, abnormal blood rheology, and abnormal expression of cytokines [13, 16]. DN's most frequent influencing variables are hypertension and hyperglycemia, with increased platelet adhesion and aggregation, reduced red blood cell deformability, and increased blood viscosity playing a larger role [17]. It was believed that effective antihypertensive, hypoglycemic, lipid regulation, and dietary control could delay DN's progression and may reverse the course of DN and improve the the prognosis of patients [18]. In this study, the treatments as mentioned earlier were given for comparison to analyze the value of hydroxychloroquine and Huangqi tablets.

Patients with DN are often accompanied by metabolic syndrome, which manifests as hypertension, hyperglycemia, and hyperlipidemia, which will deepen the degree of DN, so the treatment should focus on controlling blood pressure, glucose, and lipid [19]. The results of this study showed that, after 3 months of treatment, glycemic indices FPG, 2-hour PG, and HbA1c, as well as TC and TG levels, were all lower in group B than in group A, which received routine treatment combined with hydroxychloroquine. Group C, which received routine treatment alone, and the levels of each glycemic and lipid index in group A were lower than those in group C (*P* < 0.05), while the difference within group C before and after treatment was not significant (*P* > 0.05). It suggested that hydroxychloroquine therapy can control blood glucose and lipid levels more effectively. The combination of hydroxychloroquine therapy with Huangqi tablets can further improve blood glucose and lipid levels. Huangqi pills work by inducing diuresis and eliminating edema, which helps to control blood lipid levels and enhance renal microcirculation, raise plasma protein levels, and speed up insulin production. As a result, the patient's blood glucose level increases level can be improved. Huangqi tablets enable coronary and renal vasodilatation, dilate systemic peripheral blood vessels, and promote cutaneous blood flow, reducing blood pressure levels [20]. Huangqi tablets enhance glycogen synthase activity, protein kinase activity, and insulin receptor substrate activity and elevate glucose transporter protein levels in cardiac muscle tissue, increasing insulin sensitivity, and exerting better glycemic control [21].

In this study, the posttreatment renal function indexes SCR, BUN, and 24-hour urine protein were lower in group B than in groups A and C, and eGFR was higher than that in groups A and C. It indicates that the hydroxychloroquine combined Huangqi tablets can reduce SCR, BUN, 24-hour urine protein and increase eGFR more substantially than hydroxychloroquine alone, and solo routine treatment has no significant improvement effect on renal function. Hydroxychloroquine exerts immunomodulatory effects via its effects on autoimmune processes, as evidenced by its influence on autopeptide recognition and antigen presentation, inhibiting downstream cytokines and Th-1-type cellular immune responses [22]. Hydroxychloroquine has been found to delay the progression of renal disease and may improve prognosis [23]. After 6 months, patients treated with hydroxychloroquine for cancer in the trial lived substantially longer and had a reduced incidence of kidney damage [24]. Huangqi pills include astragalus saponin, astragalus polysaccharide, amino acids, and trace elements that may act as a diuretic and antiswelling agent and prevent and reverse urinary protein buildup [25]. It was confirmed that Huangqi tablets could delay fibrosis of kidney tissue and renal sclerosis and effectively protect the glomerular basement membrane barriers, thus playing a good protective effect on kidney function [26]. Huangqi tablets could promote vasodilation, increases blood flow to the kidneys, and inhibit nitric oxide secretion, thus correcting the renal hyperfiltration and hyperperfusion during early stage of DN [27]. It was found that 24-hour urine protein increases more significantly in patients with DN treated with Huangqi tablets than in those receiving routine therapy only [28]. In this study, the levels of VEGF, IGF-1, and TGF-*β*1 were lower in group B than in groups A and C after treatment, and group A was lower than group C (*P* < 0.05). Group B exhibited better control of cytokine levels because Huangqi tablets increase the expression of hepatocyte growth factor, thus inhibiting TGF-*β* expression, causing less free radical damage and increasing superoxide dismutase activity. Huangqi tablets also have a good antagonistic effect on calcium ions [29]. In this study, the total symptom score at 2, 4, and 6 months after treatment in group B was lower than that in groups A and C (*P* < 0.05). After 3 months of treatment in group A, the total effective rate was lower than that in group B. Still, both were higher than that in group C. The difference in the incidence of adverse reactions during treatment in groups A and B was not statistically significant. Still, both were higher than that in group C. These data suggested that hydroxychloroquine combined with Huangqi tablets in addition to routine therapy can more effectively control the symptoms of DN and can achieve higher efficacy. Meanwhile, via synergistic actions, it may decrease the negative effects of hydroxychloroquine and enhance treatment safety.

In conclusion, hydroxychloroquine combined with Huangqi tablets in the treatment of DN is better than hydroxychloroquine in addition to routine treatment, which has better control on blood glucose and blood lipids, can more effectively delay renal lesions and effectively inhibit the level of tethered cytokines. However, this study also has shortcomings, as demonstrated by the fact that only three groups were included, and the efficacy of routine treatment combined with Huangqi tablets was not analyzed. The mechanism of action of hydroxychloroquine on DN was not explored in-depth, which need to be improved in future studies.

## Figures and Tables

**Figure 1:** Blood glucose. FPG (a), 2-hour PG (b), and HbA1c (c) levels. ^*∗*^*P* < 0.05.

**Figure 2:** Blood lipids. TC (a) and TG (b). ^*∗*^*P* < 0.05.

**Figure 3:** Renal function. SCR (a), BUN (b), 24-hour urine protein (c). ^*∗*^*P* < 0.05.

**Figure 4:** Cytokines. VEGF (a), IGF-1 (b), and TGF-*β*1 (c). ^*∗*^*P* < 0.05.

**Figure 5:** Symptom score.

**Table 1:** Comparison of baseline data ($\bar{x}$ ± *s*)/[n(%).

Data		Group A (*n* = 27)	Group B (*n* = 27)	Group C (*n* = 26)	*t/X* ^2^	*P*
Gender	Male	13 (48.15)	15 (55.56)	14 (53.85)	1.072	0.391
	Female	14 (51.85)	12 (44.44)	12 (46.15)		

Age (years)		52.16 ± 11.76	53.65 ± 11.45	50.94 ± 12.43	1.113	0.095
BMI (kg/m^2^)		24.15 ± 1.25	25.02 ± 1.31	24.61 ± 1.29	0.768	0.225
Duration of type 2 diabetes mellitus (years)		7.15 ± 2.62	7.55 ± 2.79	7.38 ± 2.49	0.429	0.311
Duration of diabetic nephropathy (years)		0.78 ± 0.34	0.82 ± 0.29	0.84 ± 0.36	0.581	0.134

**Table 2:** Comparison of total effective rate after 3 months of treatment (*n* (%)).

Group	Markedly effective	Improved	Ineffective	Total effective rate
Group a (*n* = 27)	8 (29.63)	10 (37.04)	9 (33.33)	18 (66.67)
Group B (*n* = 27)	12 (44.44)	12 (44.44)	3 (11.11)	24 (88.89)
Group C (*n* = 26)	3 (11.54)	7 (26.92)	16 (61.54)	10 (38.46)
*X* ^2^				15.784
*P*				0.003

**Table 3:** Comparison of the incidence of adverse reactions (*n* (%)).

Group	Gastrointestinal adverse reactions	Retinal lesions	Central nervous system lesions	Dizziness	Elevated creatinine	Total incidence
Group A (*n* = 27)	4 (14.81)	2 (7.41)	2 (7.41)	1 (3.70)	1 (3.70)	10 (37.04)
Group B (*n* = 27)	3 (11.11)	0 (0.00)	0 (0.00)	2 (7.41)	2 (7.41)	7 (25.93)
Group C (*n* = 26)	2 (7.69)	0 (0.00)	0 (0.00)	1 (3.85)	0 (0.00)	3 (11.54)
*X* ^2^						6.876
*P*						0.550

## Data Availability

The data used to support the findings of this study are included within the article.
